# Gene-gene interaction network analysis of ovarian cancer using TCGA data

This article has been retracted.

**DOI:** 10.1186/1757-2215-6-88

**Published:** 2013-12-06

**Authors:** Huanchun Ying, Jing Lv, Tianshu Ying, Shanshan Jin, Jingru Shao, Lili Wang, Hongying Xu, Bin Yuan, Qing Yang

**Affiliations:** 1 Department of Gynecology and Obstetrics, Shengjing Hospital of China Medical University, No.36, Sanhao Street, Heping District, Shenyang, Liaoning Province 110004, China; 2 Department of Oncology, The fifth Hospital of Shenyang, Shenyang 110023, China; 3 Department of Gynecology and Obstetrics, The ninth Hospital of Shenyang, Shenyang 110024, China

**Keywords:** Differentially expressed genes, Function and pathway annotation, Gene-gene interaction network, Functional modules

## Abstract

**Background:**

The Cancer Genome Atlas (TCGA) Data portal provides a platform for researchers to search, download, and analysis data generated by TCGA. The objective of this study was to explore the molecular mechanism of ovarian cancer pathogenesis.

**Methods:**

Microarray data of ovarian cancer were downloaded from TCGA database, and Limma package in R language was used to identify the differentially expressed genes (DEGs) between ovarian cancer and normal samples, followed by the function and pathway annotations of the DEGs. Next, NetBox software was used to for the gene-gene interaction (GGI) network construction and the corresponding modules identification, and functions of genes in the modules were screened using DAVID.

**Results:**

Our studies identified 332 DEGs, including 146 up-regulated genes which mainly involved in the cell cycle related functions and cell cycle pathway, and 186 down-regulated genes which were enriched in extracellular region par function, and Ether lipid metabolism pathway. GGI network was constructed by 127 DEGs and their significantly interacted 209 genes (LINKERs). In the top 10 nodes ranked by degrees in the network, 5 were LINKERs. Totally, 7 functional modules in the network were selected, and they were enriched in different functions and pathways, such as mitosis process, DNA replication and DNA double-strand synthesis, lipid synthesis processes and metabolic pathways. AR, BRCA1, TFDP1, FOXM1, CDK2, and DBF4 were identified as the transcript factors of the 7 modules.

**Conclusion:**

our data provides a comprehensive bioinformatics analysis of genes, functions, and pathways which may be involved in the pathogenesis of ovarian cancer.

## Introduction

Ovarian cancer remains a significant public health burden, with the highest mortality rate of all the gynecological cancer, accounting for about three percent of all cancers in women [1]. Despite advances in surgery and chemotherapy, ovarian cancer in the majority of women will return and become resistant to further treatments [2]. Thus, identifying variations of differentially expressed genes (DEGs) will allow for the possibility of administering alternate therapies that may improve outcomes.

Bioinformatics analysis provides a first large scale integrative view of the aberrations in high grade serous ovarian cancer, with surprisingly simple mutational spectrum [3]. Previous studies have examined the role of genetic variation associated with the susceptibility, progression, treatment response, and survival of ovarian cancer [4,5]. It has been shown that high grade ovarian cancer is characterized by TP53 mutations in almost all tumors [6]. KRAS-variant is found to be a genetic marker for increased risk of developing ovarian cancer [7]. Genes related with cell cycle, lipid metabolism and cytoskeletal structure are screened as the treatment targets for ovarian cancer [8].

TCGA (The Cancer Genome Atlas) is a national collaborative program where different tumor types are being collected, and each tumor is being characterized using a variety of genome-wide platforms [9]. TCGA has recently complemented its first formal analysis of the genomic and clinical data from the ovarian carcinoma project.

In this study, we downloaded the microarray data of ovarian cancer form TCGA database for the identification of DEGs, and the annotation of abnormal functions and pathways in ovarian cancer. A gene-gene interaction (GGI) network was constructed using NetBox software, comprised by DEGs and their significant interacted genes. The network was further studied for its functional modules.

## Methods

### Gene expression profiles

We downloaded gene expression data batch8_9 from TCGA project webpage (https://tcga-data.nci.nih.gov/tcga/), including 38 ovarian cancer samples and 8 matched normal samples. Data levels are assigned for data type, platform and center in TCGA. The data we downloaded consisted of level 1–4, and we chose level 3 (for Segmented or Interpreted Data) for further study. Median method was used for the standardizations of the original data.

### Screening of DEGs

We applied the Limma package in R language, a linear regression model, to select the DEGs in ovarian cancer samples compared with the normal samples [10]. Only the genes with p-value < 0.05 and |log Fold Chance (FC)| > 1.5were screened out as DEGs.

### Functions and pathways enrichment of DEGs

The significant functions and pathways of DEGs was assessed based on the GO (Gene Ontology) [11] and KEGG (Kyoto Encyclopedia of Genes and Genomes) [12] annotations using Gestalt (Gene Set Analysis Toolkit) software. False discovery rate (FDR) less than 0.05 was set as the cut-off criteria.

### GGI network construction

The interactions between DEGs were searched using NetBox software. NetBox is a toolkit used in the establishment of interaction network based on public database of HPRD (Human Protein Reference Database) [13], Reactome [14], NCI-Nature Pathway Interaction database (PID) [15], as well as the MSKCC Cancer Cell Map [16]. Firstly, we obtained a global network. Then, DEGs were mapped onto the network, as well as the genes significantly interacted with these DEGs. Finally, we established the GGI network using the DEGs and their significant interaction nodes according to the assigned criteria (p < 0.05 and shortest path threshold was 2). We also calculate the degrees of the nodes by igraph package in R language, and identified the key nodes with high degrees.

### Functional modules analysis

Beside the GGI network under the assigned criteria, NetBox also divided the network into modules. Next, DAVID (Database for Annotation, Visualization and Integration Discovery) was used to identify the over-represented GO categories and KEGG pathways of the modules with FDR less than 0.05. DAVID could provide a high-throughput and integrated data-mining environment, and analysis gene lists derived from high-throughput genomic experiments.

## Results

### DEGs screening

The expressions profiles of the whole 46 samples included 12042 genes. By limma package, a total of 332 genes were selected as the DEGs between ovarian and normal samples, of which 146 were up-regulated.

### Significant functions and pathways of DEGs

The enriched functions and pathways of up-regulated DEGs are listed in Table 1. Functions that related to cell cycle, nucleotide binding, and mitosis of up-regulated DEGs were enriched, while cell cycle pathway was enriched. GO: 0044421 (extracellular region part) and hsa00565: Ether lipid metabolism pathway was the only enriched function and pathway of down-regulated DEGs, respectively.

**Table 1:** Significant GO terms and KEGG pathways of up-regulated DEGs

**Category**	**Term**	**Count**	**P value**	**FDR**
GOTERM_BP_FAT	GO:0007049~cell cycle	49	1.60E-28	2.58E-25
GOTERM_BP_FAT	GO:0000278~mitotic cell cycle	37	8.84E-28	1.42E-24
GOTERM_BP_FAT	GO:0022403~cell cycle phase	38	3.07E-27	4.94E-24
GOTERM_BP_FAT	GO:0000279~M phase	35	4.47E-27	7.20E-24
GOTERM_BP_FAT	GO:0007067~mitosis	29	8.44E-25	1.36E-21
GOTERM_BP_FAT	GO:0000280~nuclear division	29	8.44E-25	1.36E-21
GOTERM_BP_FAT	GO:0000087~M phase of mitotic cell cycle	29	1.41E-24	2.26E-21
GOTERM_BP_FAT	GO:0022402~cell cycle process	40	1.42E-24	2.29E-21
GOTERM_BP_FAT	GO:0048285~organelle fission	29	2.62E-24	4.22E-21
GOTERM_BP_FAT	GO:0051301~cell division	30	1.92E-22	3.09E-19
GOTERM_MF_FAT	GO:0005524~ATP binding	29	7.57E-06	0.0101086
GOTERM_MF_FAT	GO:0032559~adenyl ribonucleotide binding	29	9.78E-06	0.0130621
GOTERM_MF_FAT	GO:0030554~adenyl nucleotide binding	29	2.59E-05	0.0345973
GOTERM_MF_FAT	GO:0001883~purine nucleoside binding	29	3.42E-05	0.0456417
GOTERM_CC_FAT	GO:0015630~microtubule cytoskeleton	30	1.73E-15	2.21E-12
GOTERM_CC_FAT	GO:0005819~spindle	17	1.31E-13	1.63E-10
GOTERM_CC_FAT	GO:0044430~cytoskeletal part	31	3.05E-10	3.80E-07
GOTERM_CC_FAT	GO:0005694~chromosome	22	3.52E-10	4.38E-07
GOTERM_CC_FAT	GO:0043228~non-membrane-bounded organelle	52	9.48E-10	1.18E-06
GOTERM_CC_FAT	GO:0043232~intracellular non-membrane-bounded organelle	52	9.48E-10	1.18E-06
GOTERM_CC_FAT	GO:0044427~chromosomal part	19	5.36E-09	6.66E-06
GOTERM_CC_FAT	GO:0005856~cytoskeleton	33	1.27E-07	1.58E-04
GOTERM_CC_FAT	GO:0000793~condensed chromosome	11	1.68E-07	2.09E-04
GOTERM_CC_FAT	GO:0000777~condensed chromosome kinetochore	8	6.43E-07	7.99E-04
KEGG_PATHWAY	hsa04110:Cell cycle	17	5.33E-15	5.46E-12

GO: Gene Ontology; KEGG: Kyoto Encyclopedia of Genes and Genomes; DEGs: differentially expressed genes; BP: biological process; MF: molecular function; CC: cellular component.

### GGI network

A global network including 9264 genes and 68111 lines were obtained after the searching by NetBox. After screening, the GGI network was established (Figure 1), comprising of the selected DEGs and their interaction nodes (named as LINKER). There were 946 nodes in the network, including 209 LINKERs, 127 DEGs and 4105 lines. We calculated the degrees of the nodes in the network, and the top 10 nodes are listed in Table 2. LINKERs such as AHCTF1, B9D2, CASC5, and CCDC99 were found to be closely related with DEGs in the databases (p < 0.05).

**Figure 1:** **Gene-gene interaction network constructed by NetBox software.** The purple rhombuses are the LINKERs having the significant interactions (p < 0.05) with differentially expressed genes (DEGs), green circle are the down-regulated DEGs, and red circles are the up-regulate DEGs.

**Table 2:** Top 10 nodes in the gene-gene interaction network

**Rank**	**Node**	**Degree**	**Mark**
1	CDK2	93	ALTERED
2	AHCTF1	91	LINKER
3	APITD1	90	ALTERED
4	B9D2	90	LINKER
5	CASC5	89	LINKER
6	CCDC99	89	LINKER
7	CENPC1	85	ALTERED
8	CENPE	83	ALTERED
9	CENPH	80	ALTERED
10	CENPI	80	LINKER

Note: nodes marked as LINKER are the genes having significant interactions (p<0.05) with differentially expressed genes (DEGs), and nodes marked with ALTERED are the DEGs.

### Functional modules mining and analysis

Totally, 32 functional modules in the PPI network were given by the NetBox software, 7 of which having more than 10 genes (Figure 2). The results of functions and pathways clustering of the 7 modules are displayed in Table 3. Genes in module 1 were mainly participated in the mitosis process occurred in nucleus. Module 2 genes were mainly involved in DNA replication and DNA double-strand synthesis, affecting the enzymatic activity participated. Functions that are related with lipid synthesis processes and formation of intracellular membranes were enriched in module 3. Four cancer related pathways were enriched in module 4, and genes in this module can affect cell cycle by influencing the transcriptional function. Genes in module 6 were associated with wound healing process outside the cells. In addition, genes in module 7 were associated with some metabolic pathways, influencing the activities of proteolytic enzyme and ligase. No functions and pathways were found to be related with genes in module 5.

**Figure 2:** **Functional modules mined in the gene-gene interaction network.** The purple rhombuses are the LINKERs having the significant interactions (p < 0.05) with differentially expressed genes (DEGs), green circle are the down-regulated DEGs, and red circles are the up-regulate DEGs.

**Table 3:** Significant GO terms and KEGG pathways of the 7 functional modules

	**Category**	**Terms**	**Count**	**FDR**
Module 1	GOTERM_BP_FAT	GO:0000280~nuclear division	47	1.32E-63
	GOTERM_BP_FAT	GO:0007067~mitosis	47	1.32E-63
	GOTERM_BP_FAT	GO:0000087~M phase of mitotic cell cycle	47	3.30E-63
	GOTERM_BP_FAT	GO:0048285~organelle fission	47	1.02E-62
	GOTERM_BP_FAT	GO:0000279~M phase	48	7.59E-57
	GOTERM_CC_FAT	GO:0000775~chromosome, centromeric region	62	8.67E-113
	GOTERM_CC_FAT	GO:0000776~kinetochore	50	9.99E-95
	GOTERM_CC_FAT	GO:0000779~condensed chromosome, centromeric region	47	4.45E-91
	GOTERM_CC_FAT	GO:0000777~condensed chromosome kinetochore	44	2.07E-86
	GOTERM_CC_FAT	GO:0044427~chromosomal part	62	3.37E-77
	GOTERM_MF_FAT	GO:0008017~microtubule binding	10	2.56E-09
	GOTERM_MF_FAT	GO:0015631~tubulin binding	10	5.32E-08
	GOTERM_MF_FAT	GO:0051010~microtubule plus-end binding	5	5.00E-06
	GOTERM_MF_FAT	GO:0043515~kinetochore binding	4	1.77E-04
	GOTERM_MF_FAT	GO:0003777~microtubule motor activity	6	0.00746240
	KEGG_PATHWAY	hsa041114:Oocyte meiosis	7	1.62E-04
	KEGG_PATHWAY	hsa04110:Cell cycle	7	3.48E-04
Module 2	GOTERM_BP_FAT	GO:0005250~DNA replication	33	1.90E-52
	GOTERM_BP_FAT	GO:0006259~DNA metabolic process	34	2.23E-40
	GOTERM_BP_FAT	GO:0006261~DNA-dependent DNA replication	17	2.18E-26
	GOTERM_BP_FAT	GO:0006270~DNA replication initiation	12	7.20E-23
	GOTERM_BP_FAT	GO:0007049~cell cycle	17	6.59E-08
	GOTERM_CC_FAT	GO:0005654~nucleoplasm	32	3.08E-30
	GOTERM_CC_FAT	GO:0031981~nuclear lumen	32	1.62E-23
	GOTERM_CC_FAT	GO:0070013~intracellular organelle lumen	32	8.91E-21
	GOTERM_CC_FAT	GO:0043233~organelle lumen	32	1.80E-20
	GOTERM_CC_FAT	GO:0031974~membrane-enclosed lumen	32	3.28E-20
	GOTERM_MF_FAT	GO:0003677~DNA binding	26	6.52E-10
	GOTERM_MF_FAT	GO:0003688~DNA replication origin binding	5	1.25E-06
	GOTERM_MF_FAT	GO:0003697~single-stranded DNA binding	6	2.54E-04
	GOTERM_MF_FAT	GO:0016779~nucleotidylt ransferase activity	6	0.01510849
	GOTERM_MF_FAT	GO:0001882~nucleoside binding	15	0.01658336
	KEGG_PATHWAY	hsa03030:DNA replication	16	2.19E-23
	KEGG_PATHWAY	hsa04110:Cell cycle	19	1.62E-19
	KEGG_PATHWAY	hsa03420:Nucleotide excision repair	6	0.00369525
Module 3	GOTERM_BP_FAT	GO:0008610~lipid biosynthetic process	17	1.55E-13
	GOTERM_BP_FAT	GO:0008202~steroid metabolic process	13	1.63E-10
	GOTERM_BP_FAT	GO:0006694~steroid biosynthetic process	10	1.46E-09
	GOTERM_BP_FAT	GO:0055114~oxidation reduction	16	5.40E-08
	GOTERM_BP_FAT	GO:0016125~sterol metabolic process	9	3.23E-07
	GOTERM_CC_FAT	GO:0005783~endoplasmic reticulum	20	1.05E-10
	GOTERM_CC_FAT	GO:0005829~cytosol	20	3.57E-08
	GOTERM_CC_FAT	GO:0005789~endoplasmic reticulum membrane	10	1.70E-05
	GOTERM_CC_FAT	GO:0042175~nuclear envelope-endoplasmic reticulum network	10	2.72E-05
	GOTERM_CC_FAT	GO:0005792~microsome	9	1.12E-04
	GOTERM_MF_FAT	GO:0008395~steroid hydroxylase activity	8	7.37E-12
	GOTERM_MF_FAT	GO:0005506~iron ion binding	13	4.58E-08
	GOTERM_MF_FAT	GO:0046027~phospholipid:diacylglycerol acyltransferase activity	5	3.56E-07
	GOTERM_MF_FAT	GO:0016411~acylglycerol O-acyltransferase activity	6	5.50E-07
	GOTERM_MF_FAT	GO:0020037~heme binding	9	2.00E-06
	KEGG_PATHWAY	hsa00561:Glycerolipid metabolism	9	5.32E-07
	KEGG_PATHWAY	hsa00120:Primary bile acid biosynthesis	7	6.29E-07
	KEGG_PATHWAY	hsa00565:Ether lipid metabolism	8	2.94E-06
	KEGG_PATHWAY	hsa00564:Glycerophospholipid metabolism	8	3.56E-04
Module 4	GOTERM_BP_FAT	GO:0007049~cell cycle	14	8.67 E-12
	GOTERM_BP_FAT	GO:0051329~interphase of mitotic cell cycle	9	7.36E-11
	GOTERM_BP_FAT	GO:0051325~interphase	9	9.31E-11
	GOTERM_BP_FAT	GO:0000278~mitotic cell cycle	11	7.71E-10
	GOTERM_BP_FAT	GO:0022402~cell cycle process	12	1.00E-09
	GOTERM_CC_FAT	GO:0005654~nucleoplasm	10	4.75E-05
	GOTERM_CC_FAT	GO:0031981~nuclear lumen	10	0.00340842
	GOTERM_CC_FAT	GO:0070013~intracellular organelle lumen	10	0.01893931
	GOTERM_CC_FAT	GO:0043233~organelle lumen	10	0.02288144
	GOTERM_CC_FAT	GO:0031974~membrane-enclosed lumen	10	0.02691056
	GOTERM_MF_FAT	GO:0016563~transcription activator activity	7	3.96E-04
	KEGG_PATHWAY	hsa04110:Cell cycle	13	2.04 E-15
	KEGG_PATHWAY	hsa05222:Small cell lung cancer	9	8.99E-09
	KEGG_PATHWAY	hsa05200:Pathways in cancer	11	7.11E-07
	KEGG_PATHWAY	hsa05220:Chronic myeloid leukemia	7	1.89E-05
	KEGG_PATHWAY	hsa05215:Prostate cancer	7	5.34E-05
Module 6	GOTERM_BP_FAT	GO:0009511~response to wounding	9	7.88E-06
	GOTERM_BP_FAT	GO:0042060~wound healing	5	0.03445470
	GOTERM_CC_FAT	GO:0005576~extracellular region	13	2.43E-06
	GOTERM_CC_FAT	GO:0005615~extracellular space	8	0.00156546
	GOTERM_CC_FAT	GO:0044421~extracellular region part	8	0.01488625
	GOTERM_MF_FAT	GO:0005520~insulin-like growth factor binding	4	0.00208348
	GOTERM_MF_FAT	GO:0004252~serine-type endopeptidase activity	5	0.01598712
	GOTERM_MF_FAT	GO:0008236~serine-type peptidase activity	5	0.02826126
	GOTERM_MF_FAT	GO:0017171~serine hydrolase activity	5	0.02952737
	KEGG_PATHWAY	hsa:04610:Complement and coagulation cascades	4	0.03363616
Module 7	GOTERM_BP_FAT	GO:0031145~anaphase-promoting complex-dependent proteasomal ubiquitin-dependent protein catabolic process	15	1.37E-29
	GOTERM_BP_FAT	GO:0051437~positive regulation of ubiquitin-protein ligase activity during mitotic cell cycle	15	2.77E-29
	GOTERM_BP_FAT	GO:0051443~positive regulation of ubiquitin-protein ligase activity	15	4.34E-29
	GOTERM_BP_FAT	GO:0051439~regulation of ubiquitin-protein ligase activity during mitotic cell cycle	15	5.41E-29
	GOTERM_BP_FAT	GO:0051351~positive regulation of ligase activity	15	8.31E-29
	GOTERM_CC_FAT	GO:0005654~nucleoplasm	15	5.11E-13
	GOTERM_CC_FAT	GO:0005829~cytosol	16	1.27E-12
	GOTERM_CC_FAT	GO:0031981~nuclear lumen	15	5.65E-10
	GOTERM_CC_FAT	GO:0005680~anaphase-promoting complex	6	1.60E-09
	GOTERM_CC_FAT	GO:0000151~ubiquitin ligase complex	8	3.17E-09
	GOTERM_MF_FAT	GO:0004842~ubiquitin-protein ligase activity	9	1.70E-12
	GOTERM_MF_FAT	GO:0019787~small conjugating protein ligase activity	9	4.54E-12
	GOTERM_MF_FAT	GO:0016881~acid-amino acid ligase activity	9	2.17E-11
	GOTERM_MF_FAT	GO:0016879~ligase activity, forming carbon-nitrogen bonds	9	6.71E-11
	KEGG_PATHWAY	hsa04120:Ubiquitin mediated proteolysis	14	9.66E-17
	KEGG_PATHWAY	hsa04114:Oocyte meiosis	13	1.07E-15
	KEGG_PATHWAY	hsa04110:Cell cycle	13	5.29E-15
	KEGG_PATHWAY	hsa04914:Progesterone-mediated oocyte maturation	12	9.39E-15

GO: Gene Ontology; KEGG: Kyoto Encyclopedia of Genes and Genomes; FDR: false discovery rate; BP: biological process; MF: molecular function; CC: cellular component.

Besides module 7, the other 6 modules all had the down-regulated genes, such as CETN2 and CDKN1A. These genes might be suppressed in the tumorgenesis of ovarian cancer, and the biological functions and processes of them might be alternated by other promoted genes.

In all, 6 TFs were identified in the 7 modules using TRANSFAC: FOXM1 in module 1; CDK2 and DBF4 in module 2; AR, BRCA1, and TFDP1 in module 4. We got another 36 adjusted cancer-related TFs by searching TRED database.

## Discussion

Ovarian is the most lethal of all reproductive system cancers and presents a real challenge. In order to explore the molecular mechanism of ovarian cancer pathogenesis, we downloaded the gene expression profiles of ovarian cancer in the TCGA database. In the selected 332 DEGs, 146 were up-regulated genes and 186 were down-regulated genes. Cell cycle related functions, such as mitotic cell cycle and M phase; nucleotide binding related functions, such as adenyl ribonucleotide binding and purine nucleoside binding; mitosis related functions, included spindle and chromosome, and cell cycle pathway was enriched of up-regulated DEGs. In accordance with the study of Wan et al. that the up-regulated genes of ovarian carcinogenesis are related to cell cycling functions [17]. GO: 0044421 (extracellular region part) and hsa00565: Ether lipid metabolism pathway was the only enriched function pathway of down-regulated DEGs, respectively. Thus, we could infer that it is the changes of the related functions and pathways that caused the tumorgenesis of the ovarian cancer.

There were 209 LINKERs out of 336 nodes in the GGI network, as well as 5 LINKER genes in the top10 genes with high degrees in the network. LINKERs are the genes which were not identified to be abnormally expressed in ovarian cancer, but significantly interacted with the DEGs. LINKERs, such as AHCTF1, B9D2, CASC5, and CCDC99 were screened based on the literatures recorded in HPRD, Reactome, PID Interaction and MSKCC Cancer Cell Map, and they were genes in module 1. These LINKERs participated indirectly in the tumorgenesis and development of ovarian cancer by the interaction with DEGs. The abundance of LINKERs in the GGI network proved the complications of interactions between genes in ovarian cancer. AHCTF1, also known as Elys/AKNA, is originally identified as a putative transcription factor involved in mouse haematopoiesis [18]. AHCTF1 is up-regulated in ductal breast carcinomas [19], and is reported to be a risk factor for cervical cancer [20]. Mutations in B9D2 (B9 protein domain 2) has been linked to human genetic diseases [21]. CASC5 (cancer sensitibity candidate 5) has been shown to be expressed in many human cancer cell lines and in several primary human tumors [22], and CASC5 Note MLL gene and D40 gene are reported to be translocated each other in three cases of leukemia [23]. CCDC99 (coiled-coil domain containing 99) is predicted to be a mitotic spindle protein, and is over-expressed in lung cancer tumor tissues [24].

Genes such as CETN2 and CDKN1A were the down-regulated genes screened in the functional modules of the GGI network. CETN2 is an X-linked gene, it is reported that the down-regulated gene of CETN2 may have tumor suppressive functions in bladder cancer [25]. Somatic alterations of CDKN1A involved in the G1 phase of the cell cycle, are the common events in neoplastic development for multiple tumor types [26]. Thus, the biological processes and pathways of these genes might be alternated by other genes in the development of ovarian cancers.

FOXM1, CDK2, DBF4, AR, BRCA1, and TFDP1 were the TFs identified in the functional modules in GGI network. FOXM1 (Forkhead box M1) is overexpressed in a majority of human tumors, and represents as an attractive therapeutic target in the fight against cancer [27]. Forkhead TFs are intimately involved in the regulation of organismal development, cell differentiation and proliferation, and the interference with FoxM1 activity is believed to contribute to the increase in mitotic errors seen in human diseases such as cancer [28]. CDK2 (cyclin-dependent kinase 2) is found to be overexpressed in ovarian tumors, and is concur with cyclin E to ovarian tumor development [29,30]. DBF4 was a TF in module 2, and DNA replication was a significant function of module 2, which is consistent with the discovery that DBF4 is involved in the initiation of DNA replication and overexpressed in human cancer cell lines and in many primary tumors compared with the matched normal tissues [31]. The relationship between the TFs AR, BRCA1 and cancer have already been confirmed in the previous studies [32-34]. TFDP1 suppresses the colorectal cancer development by reducing telomerase activity and inhibiting the apoptosis of cells [35].

In conclusion, our data provides a comprehensive bioinformatics analysis of genes and pathways which may be involved in the pathogenesis of ovarian cancer. We have found a total of 332 DEGs, and constructed the GGI interaction networks by these DEGs and their significantly interacted genes. Furthermore, we conducted functional modules analysis in the network. However, further analyses are still required to unravel their mechanism in the process of tumor genesis and development in ovarian cancer.

## Abbreviations

DEGs: Differentially expressed genes; TCGA: The cancer genome atlas; GGI: Gene-gene interaction; GO: Gene ontology; KEGG: Kyoto encyclopedia of genes and genomes; FDR: False discovery rate; HPRD: Human protein reference database; PID: Pathway Interaction database; DAVID: Database for annotation, visualization and integration discovery; CCDC99: Coiled-coil domain containing 99; FOXM1: Forkhead box M1; CDK2: Cyclin-dependent kinase 2.

## Competing interests

The authors declare that they have no competing interests.

## Authors’ contributions

HY and HX carried out the molecular genetic studies, participated in the sequence alignment and drafted the manuscript. JL carried out the immunoassays. TY participated in the sequence alignment with LW. SJ articipated in the design of the study and performed the statistical analysis. JS, BY and QY conceived of the study, and participated in its design and coordination and helped to draft the manuscript. All authors read and approved the final manuscript.
